# Imaging of α_v_β_3_ integrin expression in experimental myocardial ischemia with [^68^Ga]NODAGA-RGD positron emission tomography

**DOI:** 10.1186/s12967-017-1245-1

**Published:** 2017-06-19

**Authors:** Maria Grönman, Miikka Tarkia, Tuomas Kiviniemi, Paavo Halonen, Antti Kuivanen, Timo Savunen, Tuula Tolvanen, Jarmo Teuho, Meeri Käkelä, Olli Metsälä, Mikko Pietilä, Pekka Saukko, Seppo Ylä-Herttuala, Juhani Knuuti, Anne Roivainen, Antti Saraste

**Affiliations:** 1 Turku PET Centre, University of Turku, 20521 Turku, Finland; 2 Heart Center, Turku University Hospital, Turku, Finland; 3 A.I.Virtanen Institute for Molecular Sciences, University of Eastern Finland, Joensuu, Finland; 4 Research Centre of Applied and Preventive Cardiovascular Medicine, University of Turku, Turku, Finland; 5 Turku PET Centre, Turku University Hospital, Turku, Finland; 6 Department of Medical Physics, Turku University Hospital and University of Turku, Turku, Finland; 7 Department of Forensic Medicine, University of Turku, Turku, Finland; 8 Turku Center for Disease Modeling, University of Turku, Turku, Finland; 9 Institute of Clinical Medicine, University of Turku, Turku, Finland

**Keywords:** Positron emission tomography, Myocardial ischemia, Angiogenesis, α_v_β_3_ integrin

## Abstract

**Background:**

Radiolabeled RGD peptides detect α_v_β_3_ integrin expression associated with angiogenesis and extracellular matrix remodeling after myocardial infarction. We studied whether cardiac positron emission tomography (PET) with [^68^Ga]NODAGA-RGD detects increased α_v_β_3_ integrin expression after induction of flow-limiting coronary stenosis in pigs, and whether α_v_β_3_ integrin is expressed in viable ischemic or injured myocardium.

**Methods:**

We studied 8 Finnish landrace pigs 13 ± 4 days after percutaneous implantation of a bottleneck stent in the proximal left anterior descending coronary artery. Antithrombotic therapy was used to prevent stent occlusion. Myocardial uptake of [^68^Ga]NODAGA-RGD (290 ± 31 MBq) was evaluated by a 62 min dynamic PET scan. The ischemic area was defined as the regional perfusion abnormality during adenosine-induced stress by [^15^O]water PET. Guided by triphenyltetrazolium chloride staining, tissue samples from viable and injured myocardial areas were obtained for autoradiography and histology.

**Results:**

Stent implantation resulted in a partly reversible myocardial perfusion abnormality. Compared with remote myocardium, [^68^Ga]NODAGA-RGD PET showed increased tracer uptake in the ischemic area (ischemic-to-remote ratio 1.3 ± 0.20, p = 0.0034). Tissue samples from the injured areas, but not from the viable ischemic areas, showed higher [^68^Ga]NODAGA-RGD uptake than the remote non-ischemic myocardium. Uptake of [^68^Ga]NODAGA-RGD correlated with immunohistochemical detection of α_v_β_3_ integrin that was expressed in the injured myocardial areas.

**Conclusions:**

Cardiac [^68^Ga]NODAGA-RGD PET demonstrates increased myocardial α_v_β_3_ integrin expression after induction of flow-limiting coronary stenosis in pigs. Localization of [^68^Ga]NODAGA-RGD uptake indicates that it reflects α_v_β_3_ integrin expression associated with repair of recent myocardial injury.

## Background

Integrins are heterodimeric transmembrane glycoprotein receptors that mediate interactions between cells and their surroundings [1, 2]. Imaging of radiolabelled arginyl-glycyl-aspartic acid (RGD) motif containing peptides targeting the α_v_β_3_ integrin has demonstrated enhanced myocardial α_v_β_3_ integrin expression after ischemic myocardial injury [3–15]. The α_v_β_3_ integrin is expressed in cardiac myofibroblasts [10, 16] and macrophages [17] involved in extracellular matrix (ECM) remodeling as well as in vascular endothelial cells during angiogenesis [3–9, 11, 13, 18], i.e. the formation of new microvascular networks from pre-existing capillaries. Since ECM remodeling and angiogenesis are essential for the healing of ischemic injury α_v_β_3_ integrin expression has been proposed as a marker of myocardial repair [3, 18]. However, it remains unknown to what extent the α_v_β_3_ integrin is expressed in response to chronic flow-limiting coronary stenosis and whether α_v_β_3_ integrin expression is induced in viable or irreversibly injured myocardium. We hypothesized that in addition to the injured myocardium ischemia induces angiogenesis and α_v_β_3_ integrin expression also in the viable ischemic myocardium.

In order to study the effects of flow-limiting coronary stenosis on myocardial expression of α_v_β_3_ integrin, we performed cardiac positron emission tomography (PET) with ^68^Gallium-labeled 1,4,7-triazacyclononane-1-glutaric acid-4,7-diacetic acid conjugated RGD peptide ([^68^Ga]NODAGA-RGD), a myocardial perfusion PET, and a histological evaluation of myocardial injury and α_v_β_3_ integrin expression in pigs. We induced stenosis by percutaneous implantation of a bottleneck stent in the proximal left anterior descending (LAD) coronary artery that has been shown to induce severe reduction in myocardial perfusion, rapid collateral formation and some degree of irreversible myocardial injury [19]. We compared [^68^Ga]NODAGA-RGD uptake in the ischemic myocardium and the remote non-ischemic myocardium as well as in the viable and injured ischemic myocardial areas 2 weeks after the induction of stenosis.

## Methods

### Animals and study protocol

Coronary stenosis was created in 11 domestic, 3-month old pigs weighing 30–35 kg by implanting a bottleneck stent in the proximal LAD coronary artery as described previously [19]. In addition, a sham group of 4 pigs underwent a catheterization procedure without the stent implantation. Myocardial [^68^Ga]NODAGA-RGD uptake was evaluated by PET 13 ± 4 days after the stent implantation. In the same imaging session, myocardial perfusion was quantified using [^15^O]water PET (physical half-life 2 min) at rest and during adenosine-induced stress before a [^68^Ga]NODAGA-RGD (physical half-life 68 min) injection to localize the myocardium and to determine the ischemic area. Three pigs without a perfusion defect during adenosine stress were considered as procedural failures and excluded from further in vivo analyses.

Subsequently, the pigs were euthanized and their hearts were excised. Based on 1% 2,3,5-triphenyltetrazolium chloride (TTC) (Sigma-Aldrich, Saint Louis, MO, USA) staining, tissue samples were obtained from the injured ischemic (TTC negative) and adjacent viable ischemic (TTC positive) myocardium as well as from the remote non-ischemic myocardium. Autoradiography of myocardial tissue sections was used to compare [^68^Ga]NODAGA-RGD uptake with the histology, α_v_β_3_ integrin expression and CD31 on endothelial cells.

### Anesthesia and hemodynamic monitoring

Prior to the cardiac catheterization and imaging studies, the animals were anesthetized with midazolam 1 mg/kg (Midazolam Hameln, Hameln Pharmaceuticals GmbH, Hameln, Germany) and xylazine 4 mg/kg (Rompun vet, Bayer Animal Health GmbH, Leverkusen, Germany) intramuscularly (i.m), connected to a respirator (Dräger Oxylog 3000, Drägerwerk AG, Lübeck, Germany) and ventilated mechanically (tidal volume 8–10 ml/kg, frequency 14–18 breaths per minute). The ear vein was cannulated using a 22G venous catheter and anesthesia was maintained with intravenous (i.v.) infusion of propofol 10–50 mg/kg/h (Propofol-Lipuro, B. Braun Melsungen AG, Melsungen, Germany) combined with fentanyl 4–8 µg/kg/h (Fentanyl-Hameln, Hameln Pharmaceuticals GmbH, Hameln, Germany). Cefuroxime (Zinacef, GlaxoSmithKline, Brentford, UK) was given 750 mg i.v. before catheterization.

The femoral artery was cannulated for hemodynamic monitoring during imaging studies. Diastolic, systolic and mean arterial pressure and heart rate were recorded using a pressure transducer (TruWave, Edwards Lifesciences, Irvine, CA, USA) connected to an anesthesia monitor.

### Coronary stenosis model

The bottleneck stent was prepared and implanted as previously described [19]. In brief, an introducer sheath (6F, Cordis, Bridgewater, NJ, USA) was placed percutaneously in the femoral artery. Catheterization of the pigs was performed in an angiographic laboratory equipped with a GE Innova 3100^IQ^ three-dimensional (3-D) angiography device (GE Healthcare, Waukesha, WI, USA). To create a coronary stenosis, a sterilized polytetrafluoroethylene tube (diameter 5/64 in.; Fluorplast, Petalax, Finland) with a bottleneck diameter of 0.9 mm was inserted on a Coroflex Blue Ultra (B. Braun Medical; profile 0.8 mm) bare metal stent. The bottleneck stent was placed into the proximal LAD. The correct positioning and patency of the bottleneck stent was confirmed by X-ray fluoroscopy, the sheath was removed and the Femostop device (St. Jude Medical, St. Paul, MN, USA) was used to secure hemostasis.

To prevent ischemia-induced arrhythmias, administration of amiodarone 200 mg/day per orally (p.o.) (Cordarone, Sanofi, Paris, France) and bisoprolol 2.5 mg/day p.o. (Bisoproact, Actavis Group, Hafnarfjordur, Island) were administered starting 1 week before the procedure until the end of the study. Immediately before stent implantation, the pigs also received a 100 mg i.v. bolus of lidocaine (Lidocain, Orion Corporation, Espoo, Finland) and 2.5 ml i.v. bolus of magnesium sulphate (246 mg/ml, Addex-magnesiumsulfaatti, Fresenius Kabi AB, Uppsala, Sweden). To prevent thrombotic occlusion of the bottleneck stent, acetylsalicylic acid 300 mg p.o. (Primaspan, Orion Corporation, Espoo, Finland) and clopidogrel 300 mg p.o. (Plavix, Sanofi, Paris, France) were given 1 day before stenting. Furthermore, enoxaparin 30 mg i.v. (Sanofi, Paris, France) was administered after the insertion of an introducer sheath in the femoral artery, and another 30 mg was given subcutaneously (s.c.) after removing the sheath and securing hemostasis. Daily doses of acetylsalicylic acid (100 mg/day p.o.), clopidogrel (75 mg/day p.o.), and enoxaparin (30 mg/day s.c.) were continued throughout the study.

### Radiochemistry

1,4,7-Triazacyclononane-1-glutaric acid-4,7-diacetic acid conjugated RGD peptide (cyclo[L-arginylglycyl-L-a-aspartyl-d-tyrosyl-N6-([[4,7-bis(carboxymethyl)-1,4,7-triazonan-1-yl]acetyl])-l-lysyl]; NODAGA-RGD) was purchased from ABX advanced biochemical compounds GmbH (product number 9805; Radenberg, Germany). ^68^Ga was obtained from a ^68^Ge/^68^Ga generator (Eckert & Ziegler, Valencia, CA, USA) by elution with 0.1 M hydrochloric acid. ^68^Ga-eluate (500 μl) was mixed with sodium acetate (18 mg) to give a pH of approximately 5. Then, NODAGA-RGD (10 nmol, dissolved in deionized water to give stock solution of 1 mM) was added. The reaction mixture was heated at 100 °C for 15 min. No further purification was performed. The radiochemical purity of [^68^Ga]NODAGA-RGD was determined by reversed-phase high-performance liquid chromatography (RP-HPLC) with a Jupiter C18 column (4.6 × 150 mm, 300 Å, 5 μm; Phenomenex, Torrance, CA, USA). The HPLC conditions were as follows: flow rate = 1 ml/min, λ **=** 220 nm. The gradient system was: A = 0.1% trifluoroacetic acid (TFA) in water; B = 0.1% TFA in acetonitrile. The A/B gradient was: 0–5 min 97/3, 5–15 min from 97/3 to 0/100. The HPLC system consisted of LaChrom Instruments (Hitachi; Merck, Darmstadt, Germany) coupled with a flow-through Radiomatic 150TR radioisotope detector (Packard, Meriden, CT, USA).

### In vitro plasma protein binding

To evaluate species-dependent differences, the [^68^Ga]NODAGA-RGD binding to human, pig and rat plasma proteins was measured using in vitro assay as described previously [20].

### PET image acquisition and reconstruction

All the animals first underwent a myocardial perfusion PET study with [^15^O]water at rest and under pharmacological stress as previously described [21] with a Discovery 690 hybrid PET/CT scanner (GE Medical Systems, Milwaukee, WI, USA). [^15^O]water (760 ± 130 MBq) was injected as an i.v. bolus over 15 s at an infusion rate of 10 ml/min via the ear vein. A dynamic acquisition of 4 min 40 s was performed (time frames 14 × 5 s, 3 × 10 s, 3 × 20 s and 4 × 30 s) in 3D mode. An adenosine infusion at the rate of 200–500 µg/kg/min combined with phenylephrine 5 µg/kg/min was started 120 s before the [^15^O]water injection and continued until the end of the scan. The acquired [^15^O]water PET data were corrected for scatter, random counts and dead time, and reconstructed with an iterative VUE Point algorithm using 2 iterations and 24 subsets. The device produces 47 axial planes with a slice thickness of 3.27 mm.

Then a [^68^Ga]NODAGA-RGD PET was performed with an ECAT EXACT HR+ scanner (Siemens-CTI, Knoxville, TN, USA). The studies were started with a 10 min transmission scan. The dynamic scanning started at the same time as 310 ± 43 MBq (230–400 MBq) of [^68^Ga]NODAGA-RGD was injected via the ear vein. The acquisition time frames were as follows: 18 × 10 s, 4 × 30 s, 2 × 120 s, 1 × 180 s, 4 × 300 s, 3 × 600 s (total duration 62 min). The acquired [^68^Ga]NODAGA-RGD PET data were corrected for scatter, random counts, and dead time and iteratively reconstructed with ordered-subsets expectation maximization (OSEM) algorithm using 2 iterations and 32 subsets. The whole transaxial field of view (70 cm) was reconstructed in 256 × 256 matrix yielding to pixel size of 2.57 mm × 2.57 mm. The device produces 63 axial planes with a slice thickness of 2.43 mm.

### PET image analysis

PET image analysis was done with Carimas 2.9 software (Turku PET Centre, Turku, Finland) using Heart and PolarRoi plug-in tools as described earlier [21, 22]. After manual definition of the long axis, the myocardial contours in the [^15^O]water images were semi-automatically defined. In order to obtain myocardial time-activity curves (TAC; the radioactivity concentrations as a function of time after the tracer injection), the PET data were volumetrically sampled and the volume of interest (VOI) covering the whole left ventricle (LV) myocardium was applied to the dynamic imaging series. The arterial input function was measured in a VOI centered in the basal part of the LV cavity. The regional LV myocardial blood flow (MBF) was quantified in [^15^O]water data as ml/min/g using a conventional single-compartment model and displayed as a parametric polar map with a standard 17 segments. The polar maps were normalized to one segment (segment 11) in the posterolateral wall that was always outside the ischemic area. The ischemic area was defined as a region with myocardial blood flow less than 80% of maximum during adenosine-induced stress as previously described [22].

For quantification of [^68^Ga]NODAGA-RGD uptake in the myocardium, the [^15^O]water images and the [^68^Ga]NODAGA-RGD images were co-registered using the high blood pool activity of the [^68^Ga]NODAGA-RGD as a landmark (Fig. 1). The myocardial contours from the [^15^O]water images were copied to the co-registered [^68^Ga]NODAGA-RGD data. Then, the polar maps of [^68^Ga]NODAGA-RGD uptake expressed as standardized uptake value (SUV) (time frame 52–62 min after injection) in the LV myocardium were generated using matching image orientation and sampling points. The region of interest (ROI) defining the ischemic area was copied from the [^15^O]water polar maps to measure [^68^Ga]NODAGA-RGD uptake in this region. The septum was excluded from the measurements to prevent spillover from the blood in the right ventricle. The mean and maximum SUVs were determined from the ischemic area. In order to measure the SUVs, ROI was modified to include only the mid-myocardium in order to avoid spill-over from blood. The maximum SUV within the ROI was determined from area showing visually the highest uptake. One segment in the posterolateral wall (segment 11) that was always outside the ischemic area was used to measure [^68^Ga]NODAGA-RGD uptake in the remote myocardium. The ischemic-to-remote SUV ratio was calculated in the ischemic area and remote myocardium.

**Fig. 1:** Co-registration of [^68^Ga]NODAGA-RGD and [^15^O]water PET images and definition of myocardial contours. **a** and **f** demonstrate [^68^Ga]NODAGA-RGD images during the first 2 min after injection of the tracer, **b** and **g** demonstrate the fusion of [^15^O]water PET images (**c**, **h**) and [^68^Ga]NODAGA-RGD images used in the co-registration (**a**, **f**). *Yellow lines* represent myocardial contours defined in [^15^O]water PET images and copied to the [^68^Ga]NODAGA-RGD images. **d** and **i** demonstrate the fusion of the [^15^O]water PET images (**c**, **h**) and [^68^Ga]NODAGA-RGD images during the last 20 min of the imaging session (**e**, **j**) that demonstrate higher activity in the ischemic area in the anteroseptal wall as compared with the remote myocardium in the inferoposterior wall

### Blood sampling and analyses

During the [^68^Ga]NODAGA-RGD PET imaging, blood samples (2 ml) were obtained into heparinized tubes from the femoral artery 2, 5, 10, 20, 30, 40, 50 and 60 min after the injection of [^68^Ga]NODAGA-RGD for the measurements of total radioactivity, radiometabolites (proportion of authentic tracer), and plasma-to-blood ratio. The radioactivities of whole blood and blood plasma were measured using a gamma counter (1480 Wizard 3″; PerkinElmer, Turku, Finland).

### Tissue sampling, autoradiography and histology

Immediately after the PET scanning, the animals were sacrificed by an i.v. injection of potassium chloride (B. Braun Medical Oy, Helsinki, Finland). The heart was excised, the LV was cut into 4 short axis slices from base to apex that were incubated for 15 min in 1% TTC (Sigma-Aldrich, Saint Louis, MO, USA), diluted in phosphate-buffered saline (pH 7.4) at 37 °C, photographed from both sides and the presence of non-viable ischemic area was confirmed visually. Based on the TTC staining, transmural samples containing non-viable and immediately adjacent viable myocardium were collected from the LV wall corresponding to the ischemic area in PET images. Another sample was obtained from the posterior LV wall representative of the remote region (segment number 11).

Myocardial samples and a blood sample were weighed and measured for radioactivity using the gamma counter (Wizard). The radioactivity concentration was expressed as standardized uptake values (SUV = ([tissue radioactivity/tissue weight]/[total given radioactivity/animal body weight])).

Tissue samples were frozen in isopentane mixed with dry ice and cut into serial 40 and 7 µm sections for autoradiography and immunohistochemical stainings respectively, using a cryomicrotome. Tissue sections of 40 μm thickness were immediately exposed on a phosphor imaging plate (BAS-TR2025, Fuji Photo Film Co. Ltd., Tokyo, Japan) for 2 h. The distribution of radioactivity on the plate was visualized and quantified using a Fluorescent Image Analyzer (Fujifilm FLA-5100, Fuji Photo Film Co. Ltd., Tokyo, Japan). Autoradiographs and hematoxylin & eosin (HE) staining images of the same sections were co-registered and [^68^Ga]NODAGA-RGD accumulation was measured by drawing ROIs covering remote myocardium, and either viable or injured ischemic myocardium using TINA™ 2.10f software (Raytest Isotopenmessgeräte GmbH., Straubenhardt, Germany). Results were expressed as photostimulated luminescence per square millimetre (PSL/mm^2^) and normalized for the injected radioactivity dose, animal weight and the radioactivity decay.

Serial tissue sections of 7 μm were stained with H&E for general histology, Masson’s trichrome for differentiation myocytes and collagenous scar, and immunohistochemistry with antibodies against of CD31 on endothelial cells (dilution 1:250, Thermo Scientific, Cheshire, UK), α_v_β_3_ integrin (dilution 1:200, Millipore, Temecula, CA, USA) and α-smooth muscle actin on myofibroblasts (dilution 1:30,000, Sigma-Aldrich, St. Louis, MO, USA). Envision (Dako, Glostrup, Denmark) and Vectastain ABC (Vector Laboratories, Burlingame, CA, USA) kits were used for detection, respectively.

### Statistical analyses

All data are expressed as mean ± SD. Statistical analysis was done with SPSS Statistics software v. 21 (IBM, NY, USA). A paired Student’s t test was applied for comparisons of the values between ischemic and remote areas. Comparisons of viable ischemic, injured ischemic and remote areas were done using ANOVA with Dunnett’s correction for remote group. A Pearson’s rank test (r) was used to analyze correlation between autoradiography and α_v_β_3_ integrin immunohistochemistry. p values less than 0.05 were considered statistically significant.

## Results

All the pigs survived the follow-up period. As shown in Fig. 2, perfusion imaging with [^15^O]water PET during adenosine stress showed a regional perfusion defect corresponding to the ischemic myocardium subtended by the stented LAD in 8 pigs that formed the final study group.

**Fig. 2:** Cardiac [^68^Ga]NODAGA-RGD and [^15^O]water in vivo PET analyses. **a** and **b** demonstrate polar maps of MBF measured by [^15^O]water PET at rest and during adenosine stress, respectively. **c** and **d** show polar maps of [^68^Ga]NODAGA-RGD uptake. Note the presence of increased [^68^Ga]NODAGA-RGD uptake in **c** co-localizing with an area of reduced myocardial perfusion (*asterisk* in **a**, **b**) as compared with the remote area (*arrowhead* in **a**, **b**). Distribution of [^68^Ga]NODAGA-RGD is homogenous in the left ventricle of sham operated pig (**d**)

### Myocardial blood flow

The average size of the ischemic area defined as MBF < 80% of the maximum during adenosine stress was 30 ± 10% of the LV as shown in Table 1. There was a regional reduction in resting perfusion within the ischemic area in 2 pigs showing reversible abnormality in the border areas. The average MBF in the ischemic area was lower than in the remote myocardium both at rest (1.4 ± 0.46 vs. 1.6 ± 0.41 ml/g/min, p = 0.0026) and during adenosine stress (1.9 ± 1.1 vs. 4.0 ± 2.2 ml/g/min, p = 0.0036). The average rate pressure product at rest and during adenosine stress was 14,000 ± 4500 and 14,000 ± 3700 mmHg bpm, respectively.

**Table 1:** Cardiac [^15^O]water and [^68^Ga]NODAGA-RGD PET

Animal	[^15^O]water PET	[^68^Ga]NODAGA-RGD PET		
	Ischemic area (% of the LV)	Remote SUV_Mean_	Ischemic area SUV_Mean_	Injured area SUV_Max_
1	19	0.68	0.71	0.95
2	17	0.37	0.56	0.67
3	35	0.52	0.70	1.11
4	32	0.47	0.56	0.74
5	19	0.36	0.54	0.72
6	36	0.65	0.79	0.94
7	37	0.42	0.41	0.59
8	43	0.45	0.57	0.70
Mean	*30*	*0.49*	0.61*	*0.80* ^†^
SD	*10*	*0.12*	*0.12*	*0.18*

The size of ischemic area based on [^15^O]water PET during adenosine stress and myocardial [^68^Ga]NODAGA-RGD uptake shown as standardized uptake value (SUV) in the remote myocardium, in the ischemic area and at the site of the highest uptake (Max) within the ischemic area

*SUV* standardized uptake value, *LV* left ventricle

* p = 0.0034 vs. remote

^†^p < 0.001 vs. remote

### Histology

In 6 pigs TTC staining showed partially injured myocardium within the ischemic area. In 4 pigs there was subendocardial injury within 1 or 2 segments, and in 2 pigs there was partially transmural injury extending to 3 segments.

Histological findings in tissue samples from the remote area and viable ischemic or injured area are described in Figs. 3 and 4. Tissue sections from the injured area showed characteristic histological features of recent ischemic myocardial injury. There was mainly loose connective tissue with some mature collagen fibers among a large amount of myofibroblasts and inflammatory cells. Viable ischemic areas showed normal distribution of myocytes and connective tissue, but some myocyte vacuolization probably related to ischemia was seen. The remote myocardium appeared histologically normal.

**Fig. 3:** Myocardial histology. *Left panel* representative image of 2,3,5-triphenyltetrazolium chloride (TTC) staining. The *arrows* show the areas where the tissue samples of the injured area, viable ischemic area and remote area were collected. **a**–**o** demonstrate stainings of hematoxylin-eosin (**a**–**c**) and Masson’s trichrome (**d**–**f**), and immunohistochemical stainings of CD31 (**g**–**i**), α_v_β_3_ integrin (**j**–**l**) and α-smooth muscle actin (**m**–**o**), and autoradiography (**p**–**r**) from the remote myocardium, from the viable ischemic area or injured myocardium based on TTC staining. *Scale bar* 50 µm

**Fig. 4:** Immunohistochemistry of endothelial cells and α_v_β_3_ integrin. The graphs in **a** and **b** show areal percentages of myocardium stained with CD31 antibodies (endothelial cells) and α_v_β_3_ integrin antibodies, respectively. Integrin α_v_β_3_ staining correlates with the [^68^Ga]NODAGA-RGD uptake measured by autoradiography in the viable ischemic area, in the injured area and in the remote area (**c**)

The immunohistochemical staining of CD31 showed positive staining in endothelial cells lining the capillaries (Fig. 3). There was no statistically significant difference in the areal percentage of the myocardium stained with CD31 between the remote myocardium and either the viable ischemic or the injured myocardium (Fig. 4).

The immunohistochemical staining of α_v_β_3_ integrin was localized around the capillaries in the viable myocardium, but also showed a diffuse distribution in the injured myocardium (Fig. 3). The areal percentage of the myocardium stained with α_v_β_3_ integrin was higher in the injured area than in the remote myocardium (23 ± 1.9% vs. 7.5 ± 1.0%, p < 0.001), but there was no difference between the viable ischemic myocardium (10 ± 4.0% vs. 7.5 ± 1.0%, p = 0.15) and the remote area (Fig. 4).

There was intense α-SMA positive staining in the injured myocardium (Fig. 3). The area of the myocardium stained with α-SMA antibody was higher in the injured than in the remote area (7.2 ± 2.9% vs. 1.3 ± 0.75%, p = 0.019).

### Radiochemical analyses and protein binding

The radiochemical purity and specific radioactivity of [^68^Ga]NODAGA-RGD were >99% and 35 ± 2.8 GBq/µmol at the end of syntheses, respectively. The tracer remained stable in vivo throughout the PET imaging with the proportion of intact tracer being >98%. The plasma-to-blood ratio of the tracer was 1.4 ± 0.10. The plasma free fraction was 0.94 ± 0.011 in the rat, 0.93 ± 0.017 in the pig and 0.91 ± 0.081 in the human serum. Thus, binding of the tracer in the plasma proteins was low in all tested species.

### [^68^Ga]NODAGA-RGD PET Imaging

Analysis of the [^68^Ga]NODAGA-RGD PET images is demonstrated in Figs. 1 and 2, and time-activity curves are shown in Fig. 5. There was virtually no tracer uptake in the normal LV myocardium and tracer activity in the blood pool remained higher than myocardial activity throughout the imaging. Based on the [^15^O]water PET images, myocardial contours were drawn in the [^68^Ga]NODAGA-RGD images to analyze regional tracer uptake. This demonstrated homogenous [^68^Ga]NODAGA-RGD distribution in sham operated pigs (coefficient of variation between segments 15 ± 6.3%), whereas uptake was regionally increased in all stented pigs within the ischemic area defined from the [^15^O]water perfusion imaging.

**Fig. 5:** Kinetics [^68^Ga]NODAGA-RGD. Mean (n = 8) time-activity curves of average [^68^Ga]NODAGA-RGD uptake in the remote myocardium, in the ischemic area and in the blood from the whole imaging session (**a**) and from the end part of the imaging session (**b**)

Mean and maximum myocardial [^68^Ga]NODAGA-RGD uptakes in the ischemic area and in the remote myocardium of stented pigs are shown in Table 1 and Fig. 6. In the ischemic area, the average myocardial [^68^Ga]NODAGA-RGD uptake was 26% higher than in the remote myocardium (p = 0.003). The maximum uptake values inside the ischemic area of the pigs were 73 and 46% higher than in the remote myocardium in pigs with viable ischemic or injured myocardium, respectively (p = 0.010 and p = 0.013, respectively, Table 1). There was no correlation between the size of the ischemic area and the amount of [^68^Ga]NODAGA-RGD uptake. The average [^68^Ga]NODAGA-RGD uptake in the LV myocardium of the sham group was similar to the remote area of the stented pigs (SUV 0.42 ± 0.10 vs. 0.49 ± 0.12 (p = 0.38) and there was no difference in the uptake between the anteroseptal (segments 7 and 13) and posterolateral (segment 11) walls in the sham group (SUV 0.39 ± 0.11 vs. 0.36 ± 0.078, p = 0.28).

**Fig. 6:** Quantification of [^68^Ga]NODAGA-RGD uptake. The graphs in **a** show [^68^Ga]NODAGA-RGD uptake measured in PET images in the remote myocardium and in the ischemic area. **b** Shows [^68^Ga]NODAGA-RGD uptake measured with a gamma counter (ex vivo biodistribution) in myocardial tissue samples obtained from the remote myocardium and from the viable ischemic area or injured myocardium based on TTC staining. **c** Shows [^68^Ga]NODAGA-RGD uptake by autoradiography in myocardial tissue sections in the remote myocardium, viable ischemic area or injured myocardium. *n* number, *SUV* standardized uptake value

### [^68^Ga]NODAGA-RGD ex vivo biodistribution

*Ex* vivo biodistribution studies (Fig. 6) showed that the radioactivity from [^68^Ga]NODAGA-RGD was higher in the tissue sample obtained from the injured myocardium (TTC negative) compared to the tissue sample obtained from the remote myocardium (SUV 0.79 ± 0.21 vs. 0.49 ± 0.21, p = 0.016), but there was no difference between the samples obtained from the remote myocardium and the viable ischemic (TTC positive) myocardium (SUV 0.49 ± 0.17, p = 0.99).

### [^68^Ga]NODAGA-RGD autoradiography

An autoradiography was performed on 6 pigs. The autoradiographs (Fig. 3) showed no [^68^Ga]NODAGA-RGD uptake in tissue sections from the remote myocardium. Uptake was also very low in the viable ischemic myocardium adjacent to the injured myocardium. In contrast, there were areas with clearly increased uptake in the sections containing injured myocardium. Quantitatively (Fig. 6), there was a statistically significant difference in the uptake between injured and remote myocardium (p = 0.006), whereas there was no difference in the uptake between viable ischemic myocardium and in the remote area (p = 0.82). The mean uptake values in the viable ischemic, remote, and injured areas were 2.2 ± 0.85, 1.8 ± 0.61 and 4.6 ± 2.1 PSL/mm^2^, respectively. The [^68^Ga]NODAGA-RGD uptake measured by autoradiography positively correlated to the area percentage of α_v_β_3_ integrin staining in the tissue sections (r_Pearson_ = 0.73, p = 0.0013) (Fig. 4).

## Discussion

The main findings of the present study are that [^68^Ga]NODAGA-RGD cardiac PET detected increased myocardial α_v_β_3_ integrin expression two weeks after induction of flow-limiting coronary stenosis in pig. In this model, α_v_β_3_ integrin expression and [^68^Ga]NODAGA-RGD uptake localized to the irreversibly injured myocardium, whereas tracer uptake was absent in viable ischemic areas. These results indicate that [^68^Ga]NODAGA-RGD is a potentially sensitive tool to detect areas of recent myocardial injury in the presence of chronic ischemia. These findings have implications in evaluation of patients with chronic ischemic heart disease in whom a mixture of viable ischemic and injured myocardium exists in the absence of transmural scar [23]. Expression of α_v_β_3_ integrin appears to play a central role in cardiac repair following myocardial infarction. A recent study showed in patients with acute myocardial infarction that α_v_β_3_ integrin targeted tracer ^18^F-fluciclatide uptake was highest in segments with improved contractile function [24]. Thus, imaging of α_v_β_3_ integrin expression may have potential to predict functional recovery upon reperfusion [24, 25] or monitor effects of therapies aimed at accelerating repair of myocardial injury.

[^68^Ga]NODAGA-RGD is a novel PET tracer for imaging α_v_β_3_ integrin expression composed of a pentacyclic peptide binding moiety Arg-Gly-Asp-D-Tyr-Lys coupled with the gallium chelating agent NODAGA. The precursor can be obtained in Good Manufacturing Practices quality from a commercial supplier and the tracer is being developed for clinical use [26]. In addition to good target specificity, studies have indicated favorable kinetics, dosimetry and safety profile [27, 28]. In previous studies, [^68^Ga]NODAGA-RGD uptake demonstrated α_v_β_3_ integrin expression in infarcted rat myocardium 1 week after coronary ligation [5]. Our study adds to the previous work by demonstrating that [^68^Ga]NODAGA-RGD cardiac PET detected α_v_β_3_ integrin expression in small, mainly subendocardial areas of myocardial injury in a model of chronic ischemia. We used a bottleneck stent model to induce persistent flow-limiting stenosis in pigs. Pig offers several advantages in comparison to rodent models as a model of translational cardiovascular research. The heart and the coronary artery system of pigs are almost identical to those of humans [29]. The size of the pig heart, which is more comparable to the size of the human heart than the heart of rodents, enables the use of clinical scanner and more reliable discrimination between the injured and ischemic myocardial areas. As shown earlier in this model, stent implantation immediately causes severe reduction in blood flow in the target coronary artery as shown by reduced fractional flow reserve, reduced myocardial blood flow during adenosine stress, and rapid collateral growth [19]. Although antithrombotic therapy was continued throughout the study to prevent stent occlusion, areas of organizing injury were detected in 6 animals. This may have been caused by insufficient compensation for reduction in myocardial perfusion by collateral formation, occlusion of a side branch by the stent, or thrombosis within the stent [19].

Repair following myocardial injury is triggered by a complex interaction of neurohormonal activation and upregulation of local paracrine signaling mechanisms that initiate restoration of capillary network through angiogenesis and extracellular matrix remodeling through macrophage accumulation and fibroblast activation. Expression of α_v_β_3_ integrin by vascular endothelial cells mediates angiogenesis, but also plays a role in regulation of macrophage inflammatory responses and myofibroblast differentiation during this process [16–18]. Thus, α_v_β_3_ integrin is a potential marker of repair following myocardial infarction. One main finding of our study is that [^68^Ga]NODAGA-RGD uptake was localized in the irreversibly damaged myocardial regions, but not in the adjacent viable myocardium within the ischemic area in this model. Increased expression of α_v_β_3_ integrin was confirmed by immunohistochemical staining, the amount of which correlated with [^68^Ga]NODAGA-RGD uptake in myocardial tissue samples. In the injured myocardium, staining of α_v_β_3_ integrin was diffuse among fibroblasts and inflammatory cells, and staining of α-SMA demonstrated myofibroblast differentiation, whereas endothelial cell staining with CD31 antibody demonstrated no difference in capillary density between remote, ischemic, and infarcted myocardium. These findings indicate that α_v_β_3_ integrin expression and [^68^Ga]NODAGA-RGD uptake reflected not only angiogenesis, but other processes related to scar formation. These findings are in line with a previous study that did not find evidence of enhanced angiogenesis or uptake of ^123^I-labelled cyclo(-Arg-Gly-Asp-D-Tyr-Lys(3-acetamido-2,6-anhydro-3-deoxy-β-d-glycero-d-gulo-heptanoic acid) (Gluco-RGD) in a pig model of myocardial hibernation induced by an ameroid constrictor [30]. Previous studies have shown RGD uptake and angiogenesis in severely hypoxic tissue [9, 12], but the severity and duration of the ischemia in the viable ischemic myocardium in our model were probably not sufficient to induce these.

We acknowledge that there are some limitations associated with our study. One of these is the fact that we did not test the effects of therapeutic angiogenesis on [^68^Ga]NODAGA-RGD uptake. Angiogenesis induced with gene therapy has previously been detected with [^123^I]-Gluco-RGD in hibernating pig myocardium, where spontaneous ischemia did not induce angiogenesis [30] and with [^18^F]-alfatide II ([^18^F]-AlF-NOTA-E[PEG_4_-c(RGDfk)]_2_) in rats after myocardial infarction [31]. Another limitation is that we used only one time point based on previous studies showing a peak in α_v_β_3_ integrin expression and RGD uptake between 1 and 4 weeks after an ischemic insult [3, 4, 6, 16]. We also acknowledge the small sample size in our study, especially relating to the autoradiography. Also the use of two different PET/CT scanners for [^15^O]water and [^68^Ga]NODAGA-RGD imaging due to logistic reasons is a limitation and might affect the accuracy of the co-registration of the images. Adenosine dose was adjusted in some pigs due to variable systemic hemodynamic responses. It has been shown that dipyridamole may provide stronger hyperemic response in the pig heart [32]. Respiratory and cardiac motion may affect sensitivity of [^68^Ga]NODAGA-RGD due to activity in the closely associated blood pool. Myocardial [^68^Ga]NODAGA-RGD uptake was studied at 50-60 min after injection, when blood levels were lower than 5% of their peak. Consistent with previous studies [24], [^68^Ga]NODAGA-RGD radioactivity remained higher in the blood than in the normal myocardium. In order to avoid spill over from the right ventricle influencing our results we included only segments in the mid-anterolateral and posterior wall into the in vivo PET analysis. Integrin α_v_β_3_ can be found on platelets, albeit in low concentrations [33]. Platelet count in pigs is much higher than that of humans [34] that might result in higher blood radioactivity in pigs than in human. However, we did not find any species differences in the binding of the tracer to plasma proteins between pigs, rats and humans.

## Conclusions

[^68^Ga]NODAGA-RGD cardiac PET demonstrates increased myocardial α_v_β_3_ integrin expression in a pig model of coronary stenosis. Increased α_v_β_3_ integrin expression is localized in the irreversibly injured myocardium, whereas it is absent in viable myocardium within the ischemic area. [^68^Ga]NODAGA-RGD PET may be useful for the identification of α_v_β_3_ integrin activation associated with repair of myocardial injury in the presence of coronary stenosis.

## Abbreviations

RGD: arginyl-glycyl-aspartic acid
ECM: extracellular matrix
PET: positron emission tomography
NODAGA: 1,4,7-triazacyclononane-1-glutaric acid-4,7-diacetic acid
LAD: left anterior descending coronary artery
TTC: 2,3,5-triphenyltetrazolium chloride
RP-HPLC: high-performance liquid chromatography
TFA: trifluoroacetic acid
TAC: time-activity curve
VOI: volume of interest
LV: left ventricle
MBF: myocardial blood flow
SUV: standardized uptake value
ROI: region of interest
HE: hematoxylin & eosin
PSL: photostimulated luminescence
Gluco-RGD: cyclo(-Arg-Gly-Asp-D-Tyr-Lys(3-acetamido-2,6-anhydro-3-deoxy-β-D-glycero-D-gulo-heptanoic acid)
